# Model Averaging for Improving Inference from Causal Diagrams

**DOI:** 10.3390/ijerph120809391

**Published:** 2015-08-11

**Authors:** Ghassan B. Hamra, Jay S. Kaufman, Anjel Vahratian

**Affiliations:** 1 Department of Environmental and Occupational Health, Drexel University School of Public Health, Philadelphia, PA 19104, USA; 2 Department of Epidemiology, Biostatistics, and Occupational Health, McGill University, Montreal, QC H3A 1A2, Canada; E-Mail: jay.kaufman@mcgill.ca; 3 Department of Obstetrics and Gynecology, University of Michigan, Ann Arbor, MI 48109, USA; E-Mail: amv@umich.edu

**Keywords:** model averaging, causal diagrams, directed acyclic graphs, wish bias

## Abstract

Model selection is an integral, yet contentious, component of epidemiologic research. Unfortunately, there remains no consensus on how to identify a single, best model among multiple candidate models. Researchers may be prone to selecting the model that best supports their *a priori*, preferred result; a phenomenon referred to as “wish bias”. Directed acyclic graphs (DAGs), based on background causal and substantive knowledge, are a useful tool for specifying a subset of adjustment variables to obtain a causal effect estimate. In many cases, however, a DAG will support multiple, sufficient or minimally-sufficient adjustment sets. Even though all of these may theoretically produce unbiased effect estimates they may, in practice, yield somewhat distinct values, and the need to select between these models once again makes the research enterprise vulnerable to wish bias. In this work, we suggest combining adjustment sets with model averaging techniques to obtain causal estimates based on multiple, theoretically-unbiased models. We use three techniques for averaging the results among multiple candidate models: information criteria weighting, inverse variance weighting, and bootstrapping. We illustrate these approaches with an example from the Pregnancy, Infection, and Nutrition (PIN) study. We show that each averaging technique returns similar, model averaged causal estimates. An *a priori* strategy of model averaging provides a means of integrating uncertainty in selection among candidate, causal models, while also avoiding the temptation to report the most attractive estimate from a suite of equally valid alternatives.

## 1. Introduction

Model selection is an inherent part of epidemiologic research [1], the optimal procedure for which is still debated. There is concern that investigators tend to select and report results of models that support their *a priori* beliefs about the association between the exposure and disease of interest, which is referred to as “wish bias” or “white hat bias” [2,3,4]. A growing body of research supports directed acyclic graphs (DAGs) as the first, and sometimes last, step in etiologic disease modeling [5,6]. DAGs are specified before data analysis and, thus, aid investigators in explicating their *a priori* beliefs about causal relations among variables before seeing the results of data analysis. Unfortunately, a correctly-specified DAG is not necessarily limited to one unique adjustment set; in fact, a single DAG may support many, theoretically unbiased adjustment sets. Further, many equally defensible models may lead to different conclusions regarding the research question of interest [7]. Typically, a researcher will select one among multiple adjustment sets for risk modeling when reporting results. Thus, while DAG analysis is generally an improvement over alternative approaches to model selection, most adopters must still restrict their analysis to the selection of a single regression model.

We propose the use of model averaging as a tool to account more honestly for uncertainty between apparently valid causal models [8]. We will first provide a brief rationale for the use of model averaging; then, we will illustrate its use with an empirical example where a DAG was used for variable selection, but where there were multiple, equally valid adjustment sets available. We will show three simple approaches to combine the results of multiple adjustment sets; information criteria weighting [9], inverse variance weighting, and bootstrapping. The arguments for utilizing directed acyclic graphs (DAGs) are widely available [5,6,10,11], so we will not repeat them here.

### 1.1. Uncertainty in Causal Modeling

Specification of a DAG is an important step in identifying valid causal models. Importantly, DAGs are specified before data analysis and provide a visual summary of the investigators’ beliefs about the relationships between variables of interest. This is based on *a priori* knowledge obtained from previous research or other relevant literature. Some researchers recommend specifying and presenting DAGs for all analyses so that readers understand the assumptions made by the authors before undertaking data analysis [12].

Suppose we are interested in the relationship between some exposure (E) and disease (D) for which we have developed a DAG to characterize our subject matter knowledge about potential confounders. We will assume that there are no important effect measure modifiers of this relationship, and that the DAG is a complete and accurate reflection of the causal relations in the target population. A sufficient adjustment set can be described as a subset of variables, adjustment for which will remove confounding of the E-D relationship. Within a DAG, one may identify sufficient adjustment sets which fully adjust for confounding, but from which no element may be removed without their becoming insufficient [5]. Figure 1 provides an illustration of a relatively simple DAG for the E-D relationship, confounded by variables A and B. In this simple scenario, the researcher has a choice between three adjustment sets [7]: [A,B], [A], or [B]; all three are sufficient, and the latter two are minimally sufficient, for estimating the total effect of E to D. Implicit in the identification of sufficient adjustment sets is the observation from the DAG that each will provide an equivalent amount of control for confounding. Thus, adjustment for any of the three sets identified from Figure 1 should produce equal point estimates of the E-D relationship. Note that the variance will likely differ across these three adjustment sets and that [B] would be expected to be the most efficient estimator [13]. In practice, the equivalence of the three adjustment sets identified from Figure 1 relies on many assumptions, the most well-known of which are no residual confounding, selection, missing data, or misclassification biases; also necessary are assumptions of positivity [14], consistency [15], and no interference [16].

**Figure 1:** Simple directed acyclic graph.

Outside of simulations, it is unlikely that all sufficient adjustment sets drawn from a DAG are equally unbiased. In some cases, knowledge regarding data quality or the susceptibility of variables to bias can guide the selection of a sufficient adjustment set. In the case of Figure 1, for example, elimination of A or B, but not both, will leave one sufficient adjustment set [17]. More often, DAGs contain many covariates with complex relationships. Even in the case that knowledge of bias in the measurement of particular variables aids in exclusion of sufficient sets from further consideration, it is not atypical to be left with a choice of two or more adjustment sets that appear equally valid, but result in different estimates of the E-D relationship of interest.

### 1.2. Averaging Models to Avoid Investigator Bias

Wish (or white hat) bias occurs when an investigator is inclined to report the results of models that support an *a priori* belief about the results s/he believes to be true. The motivation for this may be financial, but may also result from the belief that certain results best serve public health goals [4]. Even when a DAG is used, model results may differ in their statistical support for an exposure disease relationship or *a priori* investigator hypothesis, leaving room for wish bias to occur.

Rather than selecting a single regression model, a researcher can instead average over multiple candidate models. This circumvents the need for an investigator to choose a single model as the best for characterizing the relationship between the exposure and outcome of interest. By restricting candidate models to those supported by a DAG, we avoid consideration of models that may induce bias in the estimation of the E-D causal relationship. Examples of this bias include over-adjustment for covariates [13], or confounding of the disease risk estimates by inducing collider-stratification bias [18].

## 2. Methods

### 2.1. Example from the PIN Study

We consider a secondary analysis of the association between pre-pregnancy BMI (exposure) and cesarean delivery (outcome) among nulliparous women with a term pregnancy in the Pregnancy, Infection, and Nutrition (PIN) study [19]. The details of this study have been documented previously [20]; thus, we provide only a brief summary here. After consideration of inclusion and exclusion criteria, the final study population consisted of 612 women; among them, 297, 115, and 200 were classified as normal weight, overweight, and obese, respectively. Of the total population, 141 women had a cesarean delivery and the remaining 471 women experienced a vaginal birth after a trial of labor.

The authors of the original article provided a DAG summarizing the potential confounders of interest in their analyses. A group of maternal characteristics were placed within a single node of the DAG; this provided a streamlined presentation, but did not allow visualization of the relationships of each these variables to others, and each other. To facilitate determination of sufficient adjustment sets, we disaggregated these variables so each has its own node, and we added arrows for the relationships of these variables to others in the DAG. Further, to aid in visualization, we remove variables that were in the original DAG but would clearly not be considered in any minimally sufficient adjustment set. Our modified DAG is presented in Figure 2.

**Figure 2:** Directed Acyclic graph to obtain an unbiased effect of pre-pregnancy weight on cesarean delivery; adapted from Vahratian *et al.* (2005). Sufficient sets from this DAG are determined using DAGGITY software.

Of the variables included in the modified DAG, those considered a necessary element of at least one minimally-sufficient adjustment set included: chronic hypertension (no = 0, yes = 1), gestational weight gain (continuous kilograms), age (continuous years), height (continuous inches), race (white = 0, black = 1, other = 2), education (<12 years = 0, 12 years = 1, >12 years = 2), and pre-eclampsia/eclampsia (no = 0, yes = 1). Finally, the variables, including exposure and outcome, were treated as they were in the original analyses [20]; that is, we did not change or apply categorization to continuous variables or previously-determined categories for any variables of interest.

### 2.2. Three Approaches for Model Averaging

The goal of averaging is to base inference on the evidence from multiple models, rather than a single, selected regression model. Many authors have provided proof of principle and simulation evidence to support and explain the methods by which results from distinct statistical models can be averaged and the benefits of model averaging [7,9,21,22]; Here, we implemented three techniques for model averaging. First, we utilized the method developed and described by Burnham and Anderson using information criteria [9]. Second, we calculated the inverse variance weighted average of the candidate models [23,24]. Finally, we conducted a simple bootstrapping approach for model averaging [25].

Information criteria, usually Akaike’s (AIC) or Bayesian (BIC), are used to determine the support for any individual model in a set of models. Weighted averaging of the exposure parameter of interest with AIC requires models to be drawn from the same dataset and, thus, have the same number of observations. When we further restricted our analyses to women with complete information on all relevant covariates, the population includes 517 women; 257, 102, and 158 were normal weight, overweight, and obese, respectively. Among this restricted group, 120 women had a cesarean delivery and the remaining 397 women experienced a vaginal birth.

We also present inverse variance weighted averages and a bootstrapping approach for model averaging. Both approaches allow calculation of confidence intervals for the averaged estimate. Using these approaches, the number of observations is not restricted to complete information, as needed for AIC weighting. The inverse variance weighted average approach weighs each model’s parameter estimate by the inverse of the variance of the causal effect estimate. Then, the standard error is weighted by the number of observations with complete information; *i.e.*, records with missing information for a covariate are excluded. For the bootstrap approach, we sample (with replacement) 1000 times. Next, each model is fit to each bootstrap replication. We combine the bootstrap parameter estimates so that the total number of values of each parameter is the number of bootstrap samples multiplied by the number of models. The mean, median, 2.5th, and 97.5th percentiles of the distribution are provided. Calculations for the AIC weights and inverse variance weight model averaged estimates are provided in the Appendix.

We utilize the MuMIn and EPI packages with R statistical software (v 3.0.2). We use Akaike’s information criteria (AIC) to average log risk estimates obtained by fitting generalized linear models; however, we should note that other information criteria, such as Bayesian (BIC), may be used with the MuMIn package. Bootstrap resampling is conducted with SAS statistical software (v9.2, Cary, NC).

## 3. Results

The parameter estimates obtained from each individual model, and the averaged estimates, are presented in the Table 1, Table 2 and Table 3. Adjustment sets are numbered in Table 1 to simplify discussion; we refer to these numbers in Table 2 and Table 3. The model averaged estimates, using AIC, for the relative risk (95% confidence interval) of cesarean delivery comparing overweight or obese women to normal weight women are 1.33 (0.86, 2.03) and 1.62 (1.09, 2.39), respectively. Results using BIC weighting were identical to AIC weighting and, thus, are not presented. The inverse variance weighted relative risks for cesarean delivery among overweight or obese women compared to normal weight women are 1.37 (0.92, 2.04) and 1.61 (1.15, 2.27), respectively. Finally, the bootstrapping approach for averaging parameter estimates results in relative risks of cesarean delivery among overweight or obese women compared to normal weight women with a median (2.5th, 97.5th percentile values) of 1.34 (0.89, 2.01) and 1.57 (1.07, 2.35); the medians are slightly attenuated compared to the means of 1.37 and 1.60 (Table 3). The averaged relative risks are similar for all three averaging methods. Table 4 presents the confidence limit ratio [26] for each averaging approach. While the inverse variance weighting approach is the most precise, the difference by averaging technique is trivial in this example.

**Table 1:** Akaike’s information weighted averages.

Adjustment Set	Covariates	Overweight *vs.* Normal		Obese *vs.* Normal			
		Risk Ratio	95% CI	Risk Ratio	95% CI	AIC	Weight
1	Chronic hypertension, gestational weight gain, maternal age, maternal education, maternal race	1.38	0.92, 2.09	1.75	1.23, 2.50	552.56	0.43
2	Chronic hypertension, maternal age, maternal education, maternal race, maternal height	1.27	0.84, 1.92	1.46	1.04, 2.08	552.74	0.39
3	Gestational weight gain, maternal age, maternal education, maternal race, pre-eclampsia/eclampsia	1.38	0.91, 2.09	1.74	1.22, 2.48	555.12	0.12
4	Maternal age, maternal education, maternal height, maternal race, pre-eclampsia/eclampsia	1.29	0.85, 1.95	1.48	1.05, 2.10	556.43	0.06
	AIC Averaged values	1.33	0.86, 2.03	1.62	1.09, 2.39		

**Table 2:** Inverse variance weighted model averages.

	Overweight *vs.* Normal		Obese *vs.* Normal	
Adjustment Set	Risk Ratio	95% CI	Risk Ratio	95% CI
1	1.41	0.93, 2.11	1.86	1.32, 2.62
2	1.35	0.92, 2.00	1.48	1.06, 2.06
3	1.38	0.91, 2.09	1.74	1.22, 2.48
4	1.33	0.89, 1.97	1.43	1.02, 2.01
**Average**	1.37	0.92, 2.04	1.61	1.15, 2.27

The total sample sizes for models 1, 2, 3, and 4 are 538, 588, 517, and 556, respectively.

**Table 3:** Bootstrap model averages.

	Overweight *vs.* Normal			Obese *vs.* Normal		
Adjustment Set	Risk Ratio		95% Interval ^†^	Risk Ratio		95% Interval ^†^
	Mean	Median		Mean	Median	
1	1.39	1.36	0.92, 2.02	1.78	1.76	1.28, 2.46
2	1.34	1.31	0.90, 1.93	1.45	1.42	1.07, 1.98
3	1.40	1.38	0.87, 2.08	1.76	1.73	1.18, 2.50
4	1.34	1.32	0.87, 1.96	1.43	1.41	1.01, 1.99
**Average**	1.37	1.34	0.89, 2.01	1.60	1.57	1.07, 2.35

**^†^** 95% Intervals represent the 2.5th and 97.5th percentile of the parameter estimates obtained by bootstrap resampling.

**Table 4:** Confidence limit ratios ^1^ for each model averaging approach.

Averaging Approach	Overweight	Obese
Akaike’s Information	2.36	2.19
Inverse Variance	2.22	1.97
Bootstrap resampling	2.26	2.20

^1^ Upper limit divided by lower limit.

Gestational weight gain is included only in adjustment sets 1 and 3, while maternal height is included only in adjustment sets 2 and 4. Thus, it appears that adjustment for maternal height induces greater attenuation of the effect of weight on cesarean delivery compared to gestational weight gain. Further, adjustment sets 1 and 2 receive more of the overall weight compared to adjustment sets 3 and 4 using the AIC weighting method. In this example, weighting by information criteria and inverse variance produced similar results.

## 4. Discussion

We have suggested three approaches to average the results of confounder adjustment sets to account for uncertainty in model selection and to avoid investigator wish bias. We propose restricting candidate models to those supported by a directed acyclic graph, which allows readers to visualize and understand the causal structure and assumptions that the investigator identified before data analysis. A benefit is that researchers need not concern themselves with selection procedures such as change-in-estimate or backwards selection approaches. We preclude adjusting for causal intermediates, over-adjustment, or inducing confounding by collider stratification bias. These potential pitfalls that arise when using only prediction as the criterion for model selection have been noted by others [27,28].

Model selection continues to be a point of contention in epidemiology. Researchers are inconsistent in their choice of best practice [8,29]. Some methodologists have recommended adjustment for all baseline covariates (*i.e.*, all variables that cannot be caused by the exposure of interest) that are known to have possible connections to the outcome [30]. However, this approach is often untenable. In fact, we attempted such an approach in this example and a full model did not converge. The use of DAGs to identify appropriate confounder adjustment has been well validated by theory [5,6] and simulation [31]. If a DAG is correctly specified, adjustment sets supported by it will provide unbiased estimates of the causal effect on disease risk of some exposure of interest. Of course, it is unlikely, or impossible, that any DAG is specified with complete certainty, and it is a strong assumption that a DAG will fully represent the data generating process. Further, missing, or unmeasured, confounders not accounted for in a DAG might suggest that no adjustment set available to the researcher will provide an unbiased estimate of the causal effect. However, DAGs, at the very least, provide the means to minimize confounder bias and plainly communicate structural assumptions to readers.

One approach presented uses information criteria to weigh the estimates from each adjustment set. This technique favors models that provide stronger prediction of the outcome. However, if there is a large volume of missing data for certain covariates, the AIC averaging approach will require ignoring a great deal of available information. The bootstrapping and inverse variance weighting approaches may be preferable because they do not have this restriction. Averaged estimates were nearly identical for all three averaging techniques in our example.

Alternative approaches for model selection and averaging certainly exist. In particular, Bayesian model averaging is a popular, and well validated, approach to averaging or selecting among multiple candidate models [7,22]. While a potential alternative, use of Bayesian approaches to model averaging requires the specification of *a priori* values for all covariates considered in the procedure. This can be very helpful when there is prior information available to the researcher. However, in the absence of highly informative prior information, Bayesian model averaging may be more complicated than is necessary.

As with any approach based on DAGs, our analyses are reliant on correct specification of the causal diagram. Further, our approach does not overcome limitations of misclassification, selection bias, or residual confounding. However, *a priori* knowledge of whether any specific covariates are subject to bias, such as misclassification, can help guide selection of models for consideration when conducting model averaging. In addition, investigators should be wary of averaging non-collapsible causal estimates such as odds ratios and hazard ratios, which will, in general, differ across alternative confounder adjustment sets [32].

## 5. Conclusions

Model selection is an inherent part of any epidemiological analysis; however, investigator wish bias may unduly influence the selection of results that are reported in epidemiology. DAGs are an indispensable tool for identifying unbiased estimates of causal effect due to some exposure of interest that are established before data analyses. DAGs do not provide a means of selecting one among multiple, sufficient adjustment sets. By averaging the models supported by a DAG, we take account of uncertainty in model selection by considering all models that we believe provide unbiased estimates of exposure effect.

## 1. AIC Model Averaging

The calculations information criteria weighting are provided in Burnham and Anderson (2004). We briefly summarize the components that contribute to model averaging.

The likelihood for each model is calculated as:

(1) $${∆}_{i}=AIC_{i}-AIC_{min}$$

where g_i_ models I = 1,2…R receive a value relative to the model with the smallest AIC value, or AIC_min_. This, of course, gives the model with the smallest AIC a value of zero. Next, models are given weights based on a transformation of the likelihood into a relative probability via the following formula:

(2) $$w_{i}=\frac{\text{exp}\left(\frac{-{∆}_{i}}{2}\right)}{\sum_{r=1}^{R}\text{exp}\left(\frac{-{∆}_{r}}{2}\right)}$$

The sum of individual model probabilities will equal 1. Thus, the relative weight a model receives will be dependent on the other candidate models. However, the actual likelihoods of each model are invariant to the other candidate models. The weighted variance for each parameter, θ, is calculated as:

(3) $$\hat{var}\left(\bar{\theta }\right)={\left[\overset{R}{\underset{i=1}{\sum }}w_{i}{\left[\hat{var}\left({\hat{\theta }}_{i}\text{|}g_{i}\right)+\;{\left({\hat{\theta }}_{i}-\bar{\theta }\right)}^{2}\right]}^{1/2}\right]}^{2}$$

Finally, the model averaged θ is calculated as:

(4) $$\bar{\theta }=\overset{R}{\underset{i=1}{\sum }}w_{i}{\hat{\theta }}_{i}$$

## 2. Inverse Variance Weighting

We treat the mean as an inverse variance weighted average of θ obtained from each model, g_i_, as:

(5) $$\bar{\theta }=\frac{\sum_{i}\frac{\theta_{i}}{\sigma_{i}^{2}}}{\sum_{i}\frac{1}{\sigma_{i}^{2}}}$$

In order to calculate the weighted variance, $\;{\text{σ}}_{w}^{2}$, we weight each model variance by the total sample size, n, of the model, such that:

(6) $$\sigma_{w}^{2}=\frac{\sum_{i=1}^{R}\left(n_{i}-1\right)\sigma_{i}^{2}}{(\sum_{i=1}^{R}n_{i})-R}$$

## 3. Software code for recreating model averaged results for bootstrap and AIC techniques

**SAS code** 
      *********************************************************************************
      ***** Model averaging via bootstrapping
      ***** hamrag@fellows.iarc.fr
      ***** Example from PIN study (UNC, Chapel Hill)
      ***** To request PIN data, please visit:
      ***** http://www.cpc.unc.edu/projects/pin/datause
      ********************************************************************************;

	  ** Import data;
	  
      **proc****import** out=one datafile='YOUR Directory'
      dbms=csv replace; getnames=yes; **run**;

	  ** Recode variables from data so there are 0 references;
	   
      **data** one;
            set one;
            bmi = C_BMIIOM - **2**;
            medu = edu - **1**;
            height = C_INCHES - **65.04**; *Center height at mean;
			
            if ind = **0** then induction = **0**;
                  else induction = **1**;
            run;
			
        *********************************************
        ***** Bootstrap data, 1000 replications
        *********************************************;
		
        **proc****surveyselect** data=one out=pinboot
            seed = **280420141**
            method = urs
            samprate = **100**
            outhits
            rep = **1000**;
        **run**;
		
		
        *****************************************************************
        ***** Fit 4 minimally sufficient models, output data from each
        *****************************************************************;
		
        * Model 1: adjust: hypertension, gestational weight gain, maternal age/edu/race;
        ods output ParameterEstimates = m1out;
        **proc****genmod** data=pinboot desc;
            by Replicate;
            class bmi(ref=first);
            model cesarean = bmi hyper C_WTGAIN mom_age medu race /dist=binomial link=log;
        **run**;
		
        * Model 2: adjust: hypertension, maternal age/edu/race/height;
        ods output ParameterEstimates = m2out;
        **proc****genmod** data=pinboot desc;
            by Replicate;
            class bmi(ref=first);
            model cesarean = bmi hyper mom_age medu race height/dist=binomial link=log;
        **run**;
		
        * Model 3: adjust: gestational weight gain, maternal age/edu/race, eclampsia;
        ods output ParameterEstimates = m3out;
        **proc****genmod** data=pinboot desc;
            by Replicate;
            class bmi(ref=first);
            model cesarean = bmi C_WTGAIN mom_age medu race eclamp/dist=binomial link=log;
        **run**;
		
        * Model 4: adjust: maternal age/edu/race/height, eclampsia;
        ods output ParameterEstimates = m4out;
        **proc****genmod** data=pinboot desc;
            by Replicate;
            class bmi(ref=first);
            model cesarean = bmi mom_age medu race height eclamp/dist=binomial link=log;
        **run**;
		
		
        **********************************************
        ****Extract BMI values from each dataset
        ****First, for overweight vs normal
        **********************************************;
		
        **data** m1over (keep = Estimate Replicate model);
            set m1out;
            if Parameter = 'bmi' AND Level1 = **1**;
            model = **1**;
            run;
			
        **data** m2over (keep = Estimate Replicate model);
            set m2out;
            if Parameter = 'bmi' AND Level1 = **1**;
            model = **2**;
            run;
			
        **data** m3over (keep = Estimate Replicate model);
            set m3out;
            if Parameter = 'bmi' AND Level1 = **1**;
            model = **3**;
            run;
			
        **data** m4over (keep = Estimate Replicate model);
            set m4out;
            if Parameter = 'bmi' AND Level1 = **1**;
            model = **4**;
            run;
			
			
        **** Pool datasets and summarize estimate;
        **data** over;
            set m1over m2over m3over m4over;
            exp = exp(Estimate);
            run;
			
        *summary of bootstrap estimates by adjustment set;
        **proc****univariate** data=over;
            by model;
            var exp; 
            output out= over1a mean=mean pctlpts = **2.5**, **50**, **97.5** pctlpre=ci;
        **run**;
		
		
        *Model average of overweight *versus* normal weight;
        **proc****univariate** data=over;
            var exp; 
            output out= over1b mean=mean pctlpts = **2.5**, **50**, **97.5** pctlpre=ci;
        **run**;
		
		
        **********************************************
        ** Repeat above for obese *versus* normal
        *********************************************;
		
        **data** m1obese (keep = Estimate Replicate model);
            set m1out;
            if Parameter = 'bmi' AND Level1 = **2**;
            model = **1**;
            run;
			
        **data** m2obese (keep = Estimate Replicate model);
            set m2out;
            if Parameter = 'bmi' AND Level1 = **2**;
            model = **2**;
            run;
			
        **data** m3obese (keep = Estimate Replicate model);
            set m3out;
            if Parameter = 'bmi' AND Level1 = **2**;
            model = **3**;
            run;
			
        **data** m4obese (keep = Estimate Replicate model);
            set m4out;
            if Parameter = 'bmi' AND Level1 = **2**;
            model = **4**;
            run;
			
			
        **** Pool datasets and summarize estimate;
        **data** obese;
            set m1obese m2obese m3obese m4obese;
            exp = exp(Estimate);
            run;
			
        *summary of bootstrap estimates by adjustment set;
        **proc****univariate** data=obese;
            by model;
            var exp; 
            output out= obese1a mean=mean pctlpts = **2.5**, **50**, **97.5** pctlpre=ci;
        **run**;
		
        *Model average of overweight *versus* normal weight;
        **proc****univariate** data=obese;
            var exp; 
            output out= obese1b mean=mean pctlpts = **2.5**, **50**, **97.5** pctlpre=ci;
        **run**;
		
        *end of file;

        **R code**

        ###########################################################################
        ##### Multi-model inference with AIC weighting
        ###########################################################################
		
        ## Load relevant libraries and set working directory
		
        library(Epi)
        library(foreign)
        library(MuMIn)
        library(boot)
		
        setwd('Your directory')
		
        ## load and summarize data
		
        PIN <- read.csv('PIN.csv',header=T)
		
        str(PIN)
		
        ## Re-code BMI and Education so there is a zero referent
        ## also center height and record induction
		
        PIN$BMI <- PIN$C_BMIIOM - 2
        PIN$m_edu <- PIN$edu - 1 
        PIN$height <- PIN$C_INCHES - 65.04 # center height
        PIN$induction <- as.numeric(ifelse(PIN$ind==0,0,1)) # categorize induction into 0,1
		
        ####################################################
        ## Average over all minimally sufficient adjustment sets
        ####################################################
		
        ## restrict data to exclude missings. Necessary for averaging with AIC!
		
        keep <- c('cesarean','BMI','hyper','C_WTGAIN','mom_age','m_edu',
         'race','height','eclamp')
		 
        PIN1 <- na.omit(PIN[keep])
        attach(PIN1)
		
        #################################################################
        ## NOTE: some models run with reduced adjustment sets to obtain
        ## starting values that help with model convergence
        #################################################################
		
        ## model 1: hypertension, gestational weight gain, maternal age/edu/race
		
        m1a <- glm(cesarean ~ factor(BMI) + hyper + C_WTGAIN +
         mom_age + m_edu + race,
         family=binomial(link='log'))
		 
        m1 <- glm(cesarean ~ factor(BMI) + hyper + C_WTGAIN +
         mom_age + m_edu + race,
         family=binomial(link='log'))
		 
        summary(m1)
        ci.exp(m1)
		
        ## model 2: hypertension, maternal age/edu/race/height
		
        m2a <- glm(cesarean ~ factor(BMI) + hyper + mom_age + m_edu + 
         race,
         family=binomial(link='log')) 
		 
        m2 <- glm(cesarean ~ factor(BMI) + hyper + mom_age + m_edu + 
         race + height,
         family=binomial(link='log'), start=c(coef(m2a),0)) 
		 
        summary(m2)
        ci.exp(m2)
		
        ## model 3: gestational weight gain, maternal age/edu/race, eclampsia
		
        m3 <- glm(cesarean ~ factor(BMI) + C_WTGAIN + mom_age + m_edu + 
         race + eclamp,
         family=binomial(link='log')) 
		 
        summary(m3)
        ci.exp(m3)
		
		
        ## model 4: maternal age/edu/race/height, eclampsia
		
        m4a <- glm(cesarean ~ factor(BMI) + mom_age + m_edu + race + 
         eclamp,
         family=binomial(link='log')) 
		 
        m4 <- glm(cesarean ~ factor(BMI) + mom_age + m_edu + race + 
         eclamp + height,
         family=binomial(link='log'), start=c(coef(m4a),0)) 
		 
        summary(m4)
        ci.exp(m4)
		
        ## Average the results of the four models above
		
        models <- list(m1,m2,m3,m4)
		
        AIC_avg <- model.avg(models, rank=AIC, cumsum(weight)<=0.95)
		
        summary(AIC_avg)
        confint(AIC_avg)
		
        #end of file
		
